# Serum ADAM17 levels pre-antiviral therapy correlate with HIV patient immune reconstitution

**DOI:** 10.1016/j.heliyon.2024.e40734

**Published:** 2024-11-28

**Authors:** Ying Lin, Ming Chen, Xuelian Zhu, xiaoya cui, Suyu Sun, Xingzhong Hu

**Affiliations:** a Department of Clinical Laboratory Medicine, Wenzhou Central Hospital, Dingli Clinical School of Wenzhou Medical University, Wenzhou, 325000, China; b The Third Affiliated Hospital of Wenzhou Medical University, Ruian 325200, Zhejiang, China; c Dingli Clinical School of Wenzhou Medical University, Wenzhou, 325000, China; d Department of Infectious Diseases, Wenzhou Central Hospital, Dingli Clinical School of Wenzhou Medical University, Wenzhou, 325000, China; e Gynaecology and obstetrics, Wenzhou Central Hospital, Dingli Clinical School of Wenzhou Medical University, Wenzhou, 325000, China

**Keywords:** ADAM17, HIV, CD4^+^ T cells

## Abstract

**Background:**

The relationship between tumour necrosis factor (TNF) levels and disease progression is well-established. However, the impact of changes in the level of TNF hydrolase (A-disintegrin and metalloenzyme 17; ADAM17) in HIV patients remains to be fully elucidated.

**Methods:**

Between March 1 and December 31, 2017, data were collected from 64 HIV-positive individuals in Wenzhou. Based on their history of antiviral treatment at the time of enrollment, these patients were categorized into two cohorts: an antiviral-treated group and an untreated HIV group. Then, the serum ADAM17 levels of each group were measured and analysed.

**Results:**

In comparison to the antiviral-treated group and the control group, the untreated HIV group exhibited a significantly elevated serum ADAM17 level (p < 0.001). A significant negative correlation was observed between serum ADAM17 levels and CD4^+^ T cell counts in the untreated HIV group (r = −0.486, p = 0.001). ROC curve analysis revealed that the pre-treatment serum ADAM17 level in the untreated HIV group had moderate diagnostic accuracy for the AIDS stage (area under the curve: 0.703, p = 0.028). Additionally, serum ADAM17 levels were positively correlated with ADAM17 expression on the surface of leukocytes (r = 0.367, p = 0.018).

**Conclusion:**

Serum ADAM17 levels are significantly elevated in HIV patients and are correlated with disease progression and immune reconstitution.

## 1 Introduction

HIV is a global disease that poses a serious threat to human health. At the end of 2022, an estimated 39 million people were living with HIV worldwide and 29.8 million were receiving antiretroviral treatment. In 2022, there were 1.3 million new HIV infections and 630,000 AIDS-related deaths [1]. HAART, as the main treatment for AIDS, can significantly inhibit virus replication so that the patient's immune function can be rebuilt. This can extend their duration of life and improve their quality of life. However, despite HAART treatment, some patients continue to exhibit poor immune reconstitution, resulting in accelerated disease and death. Therefore, it is of great significance to predict disease progression and immune reconstitution markers in order to achieve timely adjustment of the patient's treatment regimen.

HIV-1 infection disrupts the immune system, leading to a chronic state of inflammatory activation. In response to stimulation, immune cells secrete a plethora of inflammatory factors, including tumour necrosis factor-alpha (TNF-α), which is integral to viral replication and disease progression [2]. A-disintegrin and metalloproteinase 17 (ADAM17), a key member of the ADAM superfamily, also known as TNF-α-converting enzyme (TACE), is a type I multi-domain transmembrane protein found in various human cells [3]. It predominantly cleaves the extracellular domains of transmembrane proteins via its hydrolase activity, thereby modulating signalling pathways critical in physiological processes such as development, regeneration and immunity, as well as pathological conditions such as chronic inflammation and tumourgenesis [4]. The activation of ADAM17 is essential for the cleavage and release of both TNF and its receptor (TNFR) [5].

Previous research indicates that HIV proteins, such as Nef, participate in the activation and shedding of ADAM17, facilitated through interactions with the Nef-associated kinase complex (NAKC) [6]. ADAM17 also plays a key role in HIV-1 replication in quiescent CD4^+^ T lymphocytes. Treatment with ADAM17 inhibitors eliminates the activation of resting CD4^+^ T lymphocytes and HIV-1 replication [7]. ADAM17 activity is associated with low T cell counts [8]. Thus, we hypothesize that serum ADAM17 levels are associated with HIV replication and transmission in vivo, as well as disease progression. However, few studies have reported on the dynamic changes in serum ADAM17 levels in HIV-1 patients and their relationship with HIV disease. This study aimed to clarify whether the serum ADAM17 level before treatment is associated with HIV disease progression, HAART and immune reconstitution. To this end, a sample of 64 HIV patients was analysed.

## 2 Objects and methods

### 2.1 Research objects

Between March 1, 2017, and December 31, 2017, 64 HIV patients were recruited from Wenzhou Central Hospital. The sample of HIV patients included 51 males and 13 females. For comparative analysis, a control group was established, consisting of 34 individuals (27 males and 7 females). The control group comprised individuals who were HIV-negative, had no severe underlying diseases, and were matched in terms of age and gender with the HIV-infected patients during the study period. Statistical analysis revealed no significant variations in the age and gender compositions of the patient group and the control group (Table 1).

**Table 1:** Characteristics of the study population.

	The control group	the antiviral-treated group	the untreated HIV group
n	34	25	39
Age, Median(IQR), Range, years	38(25–61)	39(24–62)	38(23–63)
Sex Male(%) Female(%)			
	27(79.4 %)	20(80.0 %)	31(79.5 %)
	7(20.6 %)	5(20.0 %)	8(20.5 %)
Treatment	–	NRTI + NNRTI/PI	–
CD4^+^T cells, Median (IQR), Range, x10^6^/L	Not determined	345	249
		(290.5–428.0)	(178.0–358.5)

NRTI:Nucleoside Reverse Transcriptase Inhibitor; NNRTI: Non-nucleoside Transcriptase Inhibitor; PI: Protease Inhibitor.

HIV patients were stratified into two groups based on their antiviral therapy history: an untreated HIV group (n = 39) and an antiviral-treated group (n = 25). The selection criteria for the antiviral-treated group included a minimum of two years of continuous treatment. The untreated HIV group comprised patients who had been diagnosed with HIV recently and had not yet started antiviral therapy. Subsequent to the commencement of antiviral therapy, the patients’ viral loads significantly decreased and became undetectable in all cases. The drug regimen primarily involved a combination of nucleoside reverse transcriptase inhibitors (NRTIs) and either protease inhibitors (PIs) or non-nucleoside reverse transcriptase inhibitors (NNRTIs). Patients without antiviral therapy were further categorized into two groups based on their CD4^+^ T cell count before treatment: a low CD4^+^ group (CD4^+^ T cell count <200/μL) and a high CD4^+^ group (CD4^+^ T cell count ≥200/μL).

Lymphocyte subsets, serum ADAM17 levels, and HIV nucleic loads were measured at the time of recruitment. Ethical approval for this study was granted by the Ethics Committee of Wenzhou Central Hospital. The research protocol was endorsed by all collaborating research centres.

### 2.2 Serum ADAM17 measurement

Five millilitres (5 mL) of venous blood was drawn and transferred into a non-anticoagulant tube. Following centrifugation at 3000 revolutions per minute for 10 min, the serum was separated and stored at −80 °C. Prior to laboratory analysis, the specimen was thawed at room temperature and thoroughly mixed. The lysis buffer was thawed at a temperature of 2–8 °C and maintained on ice for subsequent use. The serum was then combined with the lysis buffer at a 1:1 vol ratio, with a gentle mixing action performed with a pipette. Subsequently, the mixture was incubated on ice for 10 min to facilitate lysis. Then, centrifugation was performed at 4 °C and a speed of 12,000×*g* for 5 min. Subsequently, the supernatant was carefully collected for further analysis. Quantitative analysis was conducted using an Abcam's TACE Human ELISA Kit. After blocking unspecific binding with 1 % BSA in PBS for 2 h, the measurements were obtained by comparing the absorbance of the ELISA MB-530 at 450 nm with the respective standard curve. Each sample was assayed twice to ensure accuracy.

### 2.3 HIV viral load testing

Serum samples were first centrifuged at 13,000×*g* for 2 min to prevent the aspiration of precipitates or lipid layers. Then, the COBAS TaqMan HIV-1 Test reagents were equilibrated to room temperature after retrieval from storage at 2–8 °C, to ensure assay consistency. Upon initialization of the COBAS AmpliPrep and COBAS TaqMan instruments, and the AMPLILINK software, the reagents and consumables were loaded systematically into their designated positions. Sample racks were prepared with barcoded clips corresponding to S-tubes, and 1000 μl of each HIV sample and control were carefully transferred post-centrifugation. These were then loaded onto the COBAS AmpliPrep instrument, and the process was initiated via AMPLILINK software commands. The COBAS TaqMan run concluded by printing the results. Then, the used materials were disposed of, and the instruments were thoroughly cleaned and disinfected. Each step was meticulously recorded, along with the initials of the technician and the reviewer, to ensure procedural integrity and traceability.

### 2.4 Fluorescence-activated cell sorting (FACS) analysis

#### 2.4.1 Antibodies

The following antibodies were used in this study: ADAM17-Alexa Fluor@488 (Abcam, UK, catalogue number: ab196457), CD3-APC-H7 (BD, USA, catalogue number: 560275), CD4-Alexa 700 (BD, USA, catalogue number: 557882), CD8-PreCP (BD, USA, catalogue number: 557746). The isotope was IgG-Alexa Fluor@488 (Abcam, UK, catalogue number: ab199091). All antibodies were directly labelled mouse-antihuman monoclonal antibodies.

#### 2.4.2 Staining

Blood samples collected in 100 μL tubes containing EDTA as an anticoagulant, and tested within the last 24 h, were treated with a monoclonal antibody at saturation levels to stain for specific surface antigens. The samples were incubated in the dark at 25 °C for 30 min. Red blood cells (RBCs) were lysed with BD FACS lysis solution (10 min, 25 °C), followed by centrifugation at 300*g* for 5 min. The supernatant was discarded, and the tubes were blotted dry. The cells were resuspended in 200 μL of cold PBS, centrifuged again at 200 g for 5 min, and the supernatant was discarded. The tubes were blotted dry, and the cells were gently vortexed in 200 μL of cold PBS for flow cytometry analysis. Surface staining of 1000 cells was measured within 1 h using a BD FACS Canto II analyser. A gate with nucleated cells was set and the expression of ADAM17 on the surface of the nucleated cells within the gate was analysed using Flowji software.

### 2.5 Statistical analysis

The data were processed using SPSS version 24 statistical software. The data of nonnormal distribution was represented by the median (quartile value). Dunn's test was employed for multiple comparisons among the untreated group, the treated group and the control group, and Spearman's rank correlation analysis was used to assess the correlations between serum ADAM17 and HIV nucleic acid, CD4+T cell number variables. The diagnostic efficiency of serum ADAM17 for the AIDS stage was evaluated through receiver operating characteristic (ROC) curve analysis. Statistical significance was set at P < 0.05.

## 3 Results

### 3.1 Abnormal serum ADAM17 levels in HIV patients

Fig. 1 depicts the serum ADAM17 levels of the antiviral-treated HIV group, the untreated HIV group and the control group. Notably, the untreated HIV group displayed the highest serum ADAM17 level, which was significantly different from both the antiviral-treated group and the control group (p < 0.001). Conversely, no significant difference was observed between the antiviral-treated group and the control group (p > 0.05) (Fig. 1).

**Fig. 1:** The serum ADAM17 levels in three groups: the antiviral-treated group (n = 25), the untreated HIV group (n = 39) and the control group (n = 34). Differences among the antiviral-treated group, the untreated HIV group and the control group were calculated according to the Dunn's test for multiple comparisons. ADAM17: A-disintegrin and metalloenzyme 17. ∗∗∗: p < 0.001, ns: no statistical difference.

### 3.2 Correlation between serum ADAM17 levels and HIV viral loads in untreated HIV patients

Serum ADAM17 levels in the untreated HIV group were positively correlated with HIV viral loads, as depicted in Fig. 2 (r = 0.557, p < 0.001). Serum ADAM17 levels showed no significant correlation with HIV viral load in both the treatment and control groups (all P values > 0.5).

**Fig. 2:** Correlation between serum ADAM17 levels and HIV Viral load in HIV patients without antiviral therapy. The plasma ADAM17 levels is used as the abscissa, and HIV Viral load is plotted as the ordinate. Sample size: 39. ADAM17: A-disintegrin and metalloenzyme 17.

### 3.3 Correlation between serum ADAM17 levels and CD4^+^ T cell counts in untreated HIV patients

Serum ADAM17 levels in the untreated HIV group were negatively correlated with CD4^+^ T cell counts, as depicted in Fig. 3 (r = −0.486, p = 0.001).

**Fig. 3:** Correlation between serum ADAM17 levels and CD4^+^ T cell counts in HIV patients without antiviral therapy. The serum ADAM17 levels is used as the abscissa, and the count of CD4^+^ T cell is plotted as the ordinate. Sample size: 39. ADAM17: A-disintegrin and metalloenzyme 17. CD: Cell Differentiation Antigen.

### 3.4 Correlation between serum ADAM17 levels and AIDS phase in untreated HIV patients

A ROC curve was constructed to assess the diagnostic performance of serum ADAM17 levels in distinguishing between the low CD4 group (positive group) and the high CD4 group (negative group) (Fig. 4).

**Fig. 4:** The ROC curves of serum ADAM17 levels in the diagnosis of the AIDS phase. Sample size: 39. ADAM17: A-disintegrin and metalloenzyme 17. ROC: receiver operating characteristic. AUC: Area under the Curve. CI:continuous integration.

The area under the ROC curve (AUC) for serum ADAM17 levels was 0.806 [95 % confidence interval (CI): 0.666–0.946; P < 0.001]. A serum ADAM17 cutoff value of 462 pg/mL was identified as a diagnostic marker for the patient's AIDS phase.

### 3.5 Correlation between pre-antiviral therapy serum ADAM17 levels and immunologic reconstitution in HIV patients

Based on the CD4^+^ T cell counts one year post-antiviral therapy, patients in the untreated HIV group were classified into two groups: an immunologic reconstitution group and a non-reconstitution group. The criteria for immunologic reconstitution failure included: 1. a decline in the CD4^+^ T cell count to pre-therapy levels; 2. an absolute decrease of more than 30 % from the peak CD4^+^ T cell count before therapy; 3. a CD4^+^ T cell count consistently below 100 cells/μL. Successful immunologic reconstitution was defined as an increase in the CD4^+^ T cell count by at least 25 % from the pre-therapy baseline [9,10].

Of the 39 cases, 17 failed to achieve immunologic reconstitution, while 22 succeeded. The non-reconstitution group was classified as the positive group, and the reconstitution group as the negative group. A ROC curve was constructed to evaluate the efficacy of serum ADAM17 levels in predicting immunologic reconstitution success (Fig. 5). The AUC for serum ADAM17 levels was 0.723 [95 % CI: (0.554–0.893); P < 0.001]. A diagnostic cutoff value of 577 pg/mL was identified for the serum ADAM17 level.

**Fig. 5:** The ROC curves of serum ADAM17 levels in the evaluate of in predicting the success of immunologic reconstitution. Sample size: 39. ROC: receiver operating characteristic. AUC: Area under the Curve. CI:continuous integration.

### 3.6 Correlation between pre-antiviral therapy serum ADAM17 levels and the expression of ADAM17 on the surface of leukocytes

By flow cytometry, we analysed the expression of ADAM17 on the surface of leukocytes in the untreated HIV group (Fig. 6A and B). Serum ADAM17 levels in the untreated HIV group were positively correlated with the expression of ADAM17 on the surface of leukocytes, as depicted in Fig. 6 (r = 0.367, p = 0.018).

**Fig. 6:** Correlation between serum ADAM17 levels and the expression of ADAM17 on leukocyte surfaces in HIV patients without antiviral therapy. A) ADAM17-Alexa Fluor@488 was added to the grouping and then flow cytometry was performed using the FITC channel. B) The data on the left represents the proportion of leukocytes in the door to the total of cells (n = 39); The data on the right represent the proportion of ADAM17 expression on the surface of leukocytes in the door (n = 39). C) The serum ADAM17 levels is used as the abscissa, and the proportion of ADAM17 on leukocyte surfaces is plotted as the ordinate. Sample size: 39. ADAM17: A-disintegrin and metalloenzyme 17.

## 4 Discussion

This study evaluated serum ADAM17 levels across three cohorts: HIV patients receiving antiviral therapy, HIV patients without antiviral therapy, and a control group. Marked elevation in the ADAM17 level was observed in the untreated HIV group. Furthermore, following a specific duration of antiviral therapy, the serum ADAM17 level in the treated HIV group was significantly reduced to a level comparable to that of the control group.

In order to reveal the intrinsic relationship between serum ADAM17 concentrations and HIV replication, correlation analysis was performed. The serum ADAM17 levels in the untreated HIV group were positively correlated with HIV viral loads, as shown in Fig. 2. This is consistent with the findings of Joseph Kononchik et al. ADAM17 can release the virus by hydrolysing functional differentiation antigens on the cell surface, which are involved in virus transmission between cells [11]. On the other hand, Jung-Hyun Lee et al. found that Nef, paxillin and Pak1/2 in HIV can increase ADAM17 secretion and activity [12]. These findings suggest that abnormally elevated serum ADAM17 levels in HIV patients are associated with viral replication.

ADAM17 binds to exosomes of HIV-1-infected cells and plays a key role in HIV-1 replication in quiescent CD4^+^ T lymphocytes. ADAM17 weakens resting CD4^+^ T lymphocytes against HIV infection. Treatment with ADAM17 inhibitors eliminates activation and HIV-1 replication in resting CD4^+^ T lymphocytes [7]. To investigate the intrinsic link between serum ADAM17 levels and CD4^+^ T cell counts, correlation analysis was performed in the untreated HIV group. This analysis revealed a significant negative correlation. Additionally, an evaluation of the diagnostic efficacy of serum ADAM17 levels for identifying the AIDS stage demonstrated a close association between serum ADAM17 levels and the stage of AIDS.

Existing studies have consistently shown that the timing of initiation of antiviral therapy in HIV patients is strongly associated with immune reestablishment outcomes, with baseline CD4^+^ T cell levels prior to the initiation of therapy being an important determinant [13]. The Nef protein, a crucial domain of HIV, facilitates viral replication in bystander, quiescent CD4^+^ T cells [14]. HIV spreads, replicates and causes damage within these cells via Nef [15]. Additionally, Nef modulates the activation and secretion of ADAM17 by activating tyrosine kinase Hck [16]. Consequently, serum ADAM17 levels prior to antiviral therapy may be associated with a reduction in the resting CD4^+^ T cell count due to HIV Nef, thereby influencing post-therapy immune reconstitution [17]. In this study, serum ADAM17 levels were measured before therapy and subsequent immune reconstitution one year post-treatment was evaluated in 39 antiviral-naïve patients. The findings were consistent with the hypothesis, as depicted in Fig. 4. The results of this study are inconsistent with those of Lucero A. Ramon-Luing et al. In this prior study, TNF-α and TIM-3 levels in the peripheral blood of patients with immune reconstructive inflammatory syndrome were significantly higher than in patients without immune reconstructive inflammatory syndrome, and there was no difference in the ADAM17 levels. However, in this prior study, ADAM17 levels in patients with immune reconstitution inflammatory syndrome did not decrease with the progression of HAART treatment, which supports our conclusion that ADAM17 levels are correlated with immune reconstitution in HIV patients [17].

As the HIV infection progresses, the virus prompts infected cells to discharge exosomes containing viral proteins and RNA, thereby enhancing viral spread between cells. Recent studies indicate that HIV-released exosomes carry Nef and ADAM17, triggering unstimulated cells to secrete TNF-α [12]. Research by Jung-Hyun Lee and colleagues also identified ADAM17 within serum exosomes [8]. Therefore, we hypothesized that the level of ADAM17 in serum would be correlated with the level of ADAM17 expression on the surface of white blood cells. In order to verify this hypothesis, correlation analysis was performed. The results showed a positive correlation between ADAM17 in serum and ADAM17 expression on the surface of white blood cells, indicating that increased serum ADAM17 levels may be related to the up-regulation of ADAM17 expression on the cell surface and the release of ADAM17 after HIV infection.

Several limitations of this study should be noted. Firstly, the sample was recruited from a single centre and the size of the sample was not large. Secondly, changes in the serum ADAM17 levels of the patients not undergoing antiviral therapy were not continuously monitored, and the impact of antiviral therapy on serum ADAM17 levels was not dynamically assessed. Additionally, while a correlation between ADAM17 expression on the surface of leukocytes and serum ADAM17 levels was observed, this study did not examine the differential expression across the various leukocyte types. These limitations will be addressed in future research. Despite these limitations, these findings offer valuable insights to inform future research and treatment of HIV patients.

In summary, HIV infection results in an abnormal elevation of the serum ADAM17 level, and this is closely correlated with disease progression. Antiviral therapy effectively lowers the serum ADAM17 level. This study introduces a novel perspective suggesting that HIV may facilitate viral invasion and intercellular transmission by modulating ADAM17 secretion and leveraging its hydrolysis activity.

## CRediT authorship contribution statement

**Ying Lin:** Writing – original draft, Resources, Funding acquisition. **Ming Chen:** Software, Formal analysis. **Xuelian Zhu:** Data curation, Conceptualization. **xiaoya cui:** Data curation, Conceptualization. **Suyu Sun:** Writing – review & editing, Methodology. **Xingzhong Hu:** Writing – review & editing, Resources, Project administration, Investigation.

## Funding

This work was supported by Wenzhou Science and Technology Bureau Project (No: Y20210750).

## Declaration of Competing Interest

The authors declare that they have no known competing financial interests or personal relationships that could have appeared to influence the work reported in this paper.
